# MicroRNA-145 down-regulates mucin 5AC to alleviate airway remodeling and targets EGFR to inhibit cytokine expression

**DOI:** 10.18632/oncotarget.17933

**Published:** 2017-05-16

**Authors:** Zhe Cheng, Ling-Ling Dai, Xi Wang, Liu-Qun Jia, Xiao-Gang Jing, Peng-Fei Li, Meng Liu, Huan Wang, Lin An

**Affiliations:** ^1^ Department of Respiratory and Critical Care Medicine, Institute of Clinical Medicine, The First Affiliated Hospital of Zhengzhou University, Zhengzhou 450052, P.R. China

**Keywords:** microRNA-145, epidermal growth factor receptor, mucin 5AC, airway remodeling, cytokine

## Abstract

This study aims to explore how microRNA-145 (miR-145) affects airway remodeling and cytokine expression by targeting epidermal growth factor receptor (EGFR) to regulate mucin 5AC (MUC5AC).

Mice alveolar epithelial cells (AECs) were divided into a control, blank, miR-145 mimics, mimic control, miR-145 inhibitors, inhibitor control, si-*EGFR* and miR-145 inhibitors + si-*EGFR* group. Asthma mice models with airway remodeling were induced with an Ovalbumin (OVA) solution and randomly divided into a normal, asthma, asthma + miR-145 mimics, asthma + miR-145 mimic control, asthma + si-*EGFR* or asthma + si-*EGFR* NC group. Airway remodeling degree and histomorphology was measured using hematoxylin-eosin (HE), Masson and periodic acid-Schiff (PAS) staining. Flow cytometry was used to detect Th2 and Th17 cells in peripheral blood, ELISA was used to measure inflammatory factors. qRT-PCR and western blotting was adapted to detect the expressions of EGFR and the relevant cytokines that are regulated by miR-145.

The control, miR-145 mimics and si-*EGFR* groups showed a higher expression of miR-145 and a lower expression of EGFR and cytokines than the blank, mimic control, inhibitor control and miR-145 inhibitor + si-*EGFR* groups. Mice in the asthma + miR-145 mimics and asthma + si-*EGFR* groups showed lower WAt/Pbm, WAi/Pbm and WAm/Pbm, less inflammatory cells, less airway modeling and alleviated goblet cell hyperplasia and mucus obstruction than the asthma group. Furthermore, the expressions of EGFR and cytokines of transfected cells and lung tissues were negatively related to those of miR-145. MiR-145 can down-regulate MUC5AC by negatively targeting *EGFR* and thereby relieving airway remodeling.

## INTRODUCTION

Asthma is a common chronic respiratory condition which is characterized by periods of reversible airway obstruction known as asthma shock [1]. It affects both adults and children and occurs in all populations and areas globally with varying incidence and prevalence rates [2]. In the late stages of the disease airway remodeling occurs. This may include sub-epithelial fibrosis and hypertrophy and hyperplasia of airway smooth muscle and lead to relatively irreversible narrowing of the airways [3]. Airway remodeling is considered a consequence of eosinophilic inflammation and is associated with long-term clinical outcomes [4]. Genetic and environmental factors are recognized to contribute to asthma, therefore, the implicated genes may serve as significant pathways for therapeutic intervention [5, 6].

MiRNAs play a critical role in the regulation of innate immunity and inflammation in lung diseases such as asthma [7]. It has been reported that the pathological changes of airway smooth muscle (ASM) contribute to airway remodeling during asthma. It has also been reported that an over expression of microRNA-145 (miR-145) in ASM cells significantly inhibits KLF4 and subsequently, affects downstream cytokines leading to an enhanced proliferation and migration of ASM cells *in vitro* [8]. Accumulating evidence also shows the critical effect miR-145 has on asthma and lung disease via airway remodeling [9, 10]. Mucins are high molecular weight glycol proteins at the surface of most epithelial cells which have the function of protecting and lubricating. The expressions of mucins are implied to have associations with clinicopathological findings [11]. Mucin 5AC (MUC5AC) is a major airway mucin which is primarily expressed in goblet cells. Patients with asthma have been reported to produce rich MUC5AC mucus [12]. Epidermal growth factor receptor (EGFR) is a membrane glycoprotein (170-kDa) which contains an extracellular ligand-binding domain, a transmembrane lipophilic domain and an intracellular domain with tyrosine kinase activity [13]. EGFR signaling has been reported to participate in asthma tissue repair and airway remodeling [14]. Additionally, EGFR activation and the down-regulation of miR-145 has been shown to have a relation to lung cancer [15]. It is also reported that they are localized in human bronchi goblet cells and that there is a positive correlation between EGFR and MUC5AC expression [16]. The molecular mechanism of EGFR regulating MUC5AC expression is shown in Figure 1. From it, we hypothesize that miR-145 is involved in airway remodeling via EGFR. Hence, in our study, we explore whether miR-145 can affect airway remodeling by targeting EGFR to regulate MUC5AC. We aim to discuss the effect of miR-145 on airway remodeling and cytokine expression in hope that it can be clinically applied to treat asthma.

**Figure 1:** The molecular mechanism of EGFR in the regulation of MUC5AC

## RESULTS

### MiR-145 targets EGFR

According to the prediction of the miRanda database, a targeting relationship might exist between miR-145 and EGFR (Figure 2A). According to the results of dual luciferase reporter gene assay (Figure 2B), the normal psiCHECK-2-EGFR-3′UTR-transfected cells showed a significantly decreased absorption signal when transfected with miR-145 mimics compared to those transfected with mimics control (*P* < 0.05). Nevertheless, the psiCHECK- EGFR -Mut-3′UTR transfected-cells did not show any differences in absorption signal after being transfected with miR-145 mimics or mimics control (*P* > 0.05). This result indicates that miR-145 can specifically bind to the 3′UTR region of EGFR to inhibit its activity.

**Figure 2:** Targeting relationship between miR-145 and EGFR detected by dual luciferase reporter gene assay Note: **(A)** base sequence pairing of miR-145and EGFR; **(B)** luciferase activity after cells were transfected with miR-145 and EGFR3′UTR; *, *P* < 0.05 in comparison with the mimics control group; miR-145, microRNA-145; EGFR, epidermal growth factor receptor.

### Comparison of EGFR and related cytokines expression among the control, blank, miR-145 mimics, mimic control, miR-145 inhibitors, inhibitor control, si-EGFR and miR-145 inhibitors + si-EGFR groups

The miR-145 mimics and si-*EGFR* groups had higher miR-145 expression than the blank group, while expressions of EGFR, MUC5AC, MMP-9 and TIMP-1 were significantly decreased compared to the blank group (all *P*< 0.05). However, the miR-145 inhibitors group had a decreased miR-145 expression and a significantly increased expression of EGFR, MUC5AC, MMP-9 and TIMP-1 (all *P* < 0.05). No significant differences were found among the blank, miR-145 mimic control, miR-145 inhibitor control and miR-145 inhibitors + si-*EGFR* groups (all *P*> 0.05). Compared with other groups, the control group had an increased miR-145 expression, but decreased expression of EGFR, MUC5AC, MMP-9 and TIMP-1 (Figure 3).

**Figure 3:** Comparison of expressions of EGFR and other cytokines among the control, blank, miR-145 mimics, mimic control, miR-145 inhibitors, inhibitor control, si-EGFR and miR-145 inhibitors + si-EGFR groups Note: **(A)** The expression of miR-145, EGFR and other cytokines mRNA detected by qRT-PCR; **(B)** the expressions of EGFR and other cytokines proteins detected by western blotting; **(C)** western blotting images of expressions of EGFR and other cytokines proteins in each group (four times in each group)*, *P* < 0.05 in comparison with the blank, mimic control, inhibitor control and miR-145 inhibitors + si-*EGFR* groups; miR-145, microRNA-145; EGFR, epidermal growth factor receptor; MUC5AC, mucin 5AC; MMP-9, matrix metalloproteinase-9; TIMP-1, tissue inhibitor of metalloproteinase-1; GAPDH, glyceraldehyde-3-phosphate dehydrogenase; qRT-PCR, quantitative real-time polymerase chain reaction.

### Comparison of airway remodeling degree and morphology between each group

During the entire model construction, no mice in the normal group showed any discomfort or died. Mice in the asthma, asthma + miR-145 mimic NC and asthma + si-*EGFR* NC groups showed no obvious discomfort, however, 4∼7 mice died in each group. Mice in the asthma + miR-145 mimics and asthma + si-*EGFR* groups were in good health condition, but there were 1∼2 mice deaths. All the surviving mice were identified using a pathological biopsy. Table 1 shows the parameters of airway remodeling. All the other asthma groups showed an obvious increase of WAt/Pbm, WAi/Pbm and WAm/Pbm compared with the normal group (all *P*< 0.05). There was no significant difference in WAt/Pbm, WAi/Pbm and WAm/Pbm among the asthma, asthma + miR-145 mimic NC and asthma + si-*EGFR* NC groups (all *P* > 0.05). Compared with the asthma group, the asthma + miR-145 mimics and asthma + si-*EGFR* groups showed significantly decreased WAt/Pbm, WAi/Pbm and WAm/Pbm (all *P*< 0.05).

**Table 1:** Comparison of airway remodeling related parameters among the seven groups

Group	WAt/Pbm	WAi/Pbm	WAm/Pbm
Normal	11.51 ± 1.12	5.92 ± 0.65	3.32 ± 0.34
Asthma	31.99 ± 1.01 ^a^	29.91 ± 1.49^a^	18.85 ± 0.89 ^a^
Asthma +miR-145 mimics	19.06 ± 1.22 ^ab^	18.34 ± 1.68 ^ab^	6.75 ± 0.92 ^ab^
Asthma + miR-145 mimics NC	32.12 ± 1.04 ^a^	30.03 ± 1.54 ^a^	18.11 ± 0.99 ^a^
Asthma + si-*EGFR*	19.01 ± 1.19^ab^	18.30 ± 1.66^e^	6.69 ± 0.93 ^ab^
Asthma + si-*EGFR* NC	33.11 ± 1.26^a^	30.39 ± 1.71^a^	18.79 ± 0.95 ^a^

Note: ^a^, *P* < 0.05 in comparison with the normal group; ^b^, *P*< 0.05 in comparison with the asthma, asthma + miRNA-145 mimic NC and asthma + si-*EGFR* NC groups; 20 mice × 6 groups; miR-145, microRNA-145;WAt, total bronchial wall area; Pbm, perimeter of basement membrane; WAi, inner wall area; WAm, smooth muscle wall area; NC, normal control; EGFR, epidermal growth factor receptor.

According to the HE staining results, the airway epithelial tissues in the normal group were smooth. There was no infiltration of inflammatory cells in the periphery of the mucosa and airway smooth muscle was not thickened. Mice in the asthma, asthma + miR-145 mimic NC and asthma + si-*EGFR* NC groups did show inflammatory cell infiltration (mainly lymphocytes and eosinocytes). There was obvious airway wall and smooth muscle thickening and lumen narrowing. In the asthma + miR-145 mimics and asthma + si-*EGFR* groups, the airway epithelial tissue was smooth and inflammatory cells decreased. The differences between the two groups were not significant. According to the Masson staining, tissue in the normal group was uniformly distributed and there was no obvious inflammatory cells infiltration or thickening of smooth muscle. In the asthma, asthma + miR-145 mimic NC and asthma + si-*EGFR* NC groups, collagenous fiber increased and the collagen area of the basement membrane expanded. The asthma + miR-145 mimics and asthma + si-*EGFR* groups showed relatively less airway remodeling. The results of the PAS staining revealed that tissues in the normal group showed no goblet cell hyperplasia or mucus obstruction. Whereas mice in the asthma, the asthma + miR-145 mimic NC and the asthma + si-*EGFR* NC groups showed goblet cell hyperplasia and mucus obstruction. However, those in the asthma + miR-145 mimics and asthma + si-*EGFR* groups had alleviated goblet cell hyperplasia and mucus obstruction (Figure 4).

**Figure 4:** Comparison of histomorphology of the lung tissues among each group detected by HE and Masson staining (× 400). Note: miR-145, microRNA-145; HE, hematoxylin-eosin; PAS, periodic acid-Schiff; EGFR, epidermal growth factor receptor; 20 mice × 6 groups.

### Comparison of proportion of Th2 and Th17 cells in peripheral blood among the normal, asthma, asthma + miR-145 mimic, asthma + miR-145 mimic NC, asthma + si-EGFR and asthma + si-EGFR NC groups

Table 2 shows the proportion of Th2 and Th17 cells in CD 4+ T cells of the peripheral blood. The asthma + miR-145 mimic and asthma + si-EGFR groups had a higher proportion of Th2 and Th17 cells in peripheral blood than the normal group, but the difference is not statistically significant (*P* > 0.05). However, the asthma + miR-145 mimic and asthma + si-EGFR groups had a remarkably decreased proportion of T h2 and Th17 cells in peripheral blood than the asthma, asthma + miR-145 mimic NC and asthma + si-EGFR NC groups (all *P* < 0.05).

**Table 2:** Comparison of proportion of Th2 and Th17 cells in peripheral blood among the normal, asthma, asthma + miR-145 mimic, asthma + miR-145 mimic NC, asthma + si-EGFR and asthma + si-EGFR NC groups

Group	Th2 cell (%)	Th17 cell (%)
Normal	0.53 ± 0.19	0.92 ± 0.28
Asthma	0.91 ± 0.23*	3.54 ± 0.61*
Asthma + miR-145 mimics	0.64 ± 0.12^#^	0.99 ± 0.26^#^
Asthma + miR-145 mimics NC	0.96 ± 0.18*	3.45 ± 0.29*
Asthma + si-EGFR	0.69 ± 0.21^#^	1.09 ± 0.31^#^
Asthma + si-EGFR NC	0.92 ± 0.16*	3.29 ± 0.51*

Note: *, *P* < 0.05 in comparison with the normal control group; ^#^, *P* < 0.05 in comparison with the asthma, asthma + miR-145 mimics NC and asthma + si-EGFR NC groups; miR-145, microRNA-145; EGFR, epidermal growth factor receptor.

### Comparison of miR-145, EGFR and cytokines among the normal, asthma, asthma + miR-145 mimic, asthma + miR-145 mimic NC, asthma + si-EGFR and asthma + si-EGFR NC groups

The other groups showed significantly different expressions of miR-145, EGFR and related cytokines to the normal group. The normal group had the highest expression of miR-145 but the lowest expression of EGFR, MUC5AC, TSLP, MMP-9, TIMP-1 and cytokines. Differences were not significant among the asthma, asthma + miR-145 mimic NC and asthma + si-*EGFR* NC groups (all *P*> 0.05). Compared with the asthma group, the asthma + miR-145 mimics and asthma + si-*EGFR* groups showed significantly elevated miR-145 expression, but simultaneously reduced expressions of EGFR, MUC5AC, TSLP, MMP-9, TIMP-1 and other cytokines (all *P*< 0.05) (Figure 5 and Table 3).

**Figure 5:** Comparison of miR-145, EGFR and other cytokines expressions among the normal, asthma, asthma + miR-145 mimic, asthma + miR-145 mimic NC, asthma + si-*EGFR* and asthma + si-*EGFR* NC groups Note: **(A)**, the expressions of miR-145, EGFR and other cytokines in mice detected by qRT-PCR; **(B)**, the expressions of EGFR and other cytokines proteins in mice detected by western blotting; **(C)**, western blotting images of expressions of EGFR and other cytokines proteins in mice among each group; *, *P* < 0.05 in comparison with the normal group; #, *P* < 0.05, in comparison with the asthma, asthma + miR-145 mimic NC and asthma + si-*EGFR* NC groups; miR-145, microRNA-145; EGFR, epidermal growth factor receptor; MUC5AC, mucin 5AC; TSLP, thymic stromal lymphopoietin; MMP-9, matrix metalloproteinase-9; TIMP-1, tissue inhibitor of metalloproteinase-1; qRT-PCR, quantitative real-time polymerase chain reaction; 20 mice × 6 groups.

**Table 3:** Comparison of inflammatory cytokines in BALF among the normal, asthma, asthma + miR-145 mimic, asthma + miR-145 mimic NC, asthma + si-EGFR and asthma + si-EGFR NC groups

Group	TNF-α	IL-4	IL-5	IL-13	TSLP	IL-25	IL-33
Normal	237.44 ± 62.34	57.92 ± 12.11	77.56 ± 20.19	19.25 ± 1.23	1489 ± 22	98.45 ± 19.23	33.27 ± 10.67
Asthma	501.38 ± 153.57*	209.29 ± 54.79*	413.25 ± 110.23*	80.54 ± 7.19*	2004 ± 45*	219.78 ± 25.78*	78.56 ± 10.45*
Asthma + miR-145 mimics	301.11 ± 78.34*#	102.99 ± 32.78*#	145.79 ± 31.13*#	36.10 ± 2.11*#	1677 ± 20*#	149.04 ± 20.36*#	55.82 ± 14.29*#
Asthma + miR-145 mimics NC	516.09 ± 167.23*	200.03 ± 60.11*	411.34 ± 120.11*	81.10 ± 8.90*	2034 ± 52*	209.14 ± 20.76*	80.96 ± 12.06*
Asthma + si-EGFR	294.78 ± 67.23*#	95.53 ± 29.92*#	139.49 ± 30.11*#	37.51 ± 2.33*#	1563 ± 17*#	161.38 ± 24.06*#	74.26 ± 11.28*#
Asthma+si-EGFR NC	507.19 ± 159.26*	210.33 ± 64.89*	409.89 ± 123.78*	79.37 ± 6.48*	1701 ± 36*	202.77 ± 24.18*	60.39 ± 12.88*

Note: BALF, bronchoalveolar lavage fluid; TNF-α, tumor necrosis factor-α, IL, interleukin; TSLP, thymic stromal lymphopoietin; miR-145, microRNA-145; EGFR, epidermal growth factor receptor; *, *P* < 0.05 in comparison with the normal control;^#^, *P* < 0.05 in comparison with the asthma, asthma + miR-145 mimics NC and asthma + si-EGFR NC groups.

## DISCUSSION

Asthma is a serious health hazard worldwide and people of all ages are affected by the chronic airway disorder [17]. Making the molecular mechanism behind asthma clear would be very helpful in exploring new therapeutic targets for treatment.

In this study, we found that miR-145 targets and inhibits *EGFR* in the *EGFR*-3′UTR region. The results of the qRT-PCR and western blotting analysis confirmed that a lower expression of miR-145 causes higher EGFR. We demonstrated that MiR-145 promotes differentiation and inhibits the proliferation of smooth muscle cells [18]. The aberrant expression of EGFR is related with signaling pathways responsible for cell proliferation, invasion and metastasis in several cancers [19]. In asthma there is evidence that epithelial injury and repair are abnormal [20]. As the activation of EGFR is involved in epithelial repair after injury in damaged airway epithelium, a deregulated activation of these pathways may play an important role in remodeling in asthmatic airways [21, 22]. Bronchial epithelial EGFR expression was consistently reported to be up-regulated in patients with asthma [23, 24]. Guo YH *et al*. reported that EGFR activation is associated with the down-regulation of miR-145 in lung cancer cells [25]. Cho et al also showed that by targeting *EGFR*, miR-145 is able to inhibit human lung adenocarcinoma cell proliferation [26].

Furthermore, the study revealed that the transfection of miR-145 mimics and *EGFR* siRNA plasmid leads to an increased expression of IL-25 and a decreased expression of MUC5AC, TSLP, MMP-9 and TIMP-1. Mucus hyper-secretion is a typical symptom of asthma and excessive mucus can contribute to airflow limitation and airway obstruction [12]. EGF activates EGFR tyrosine kinases and plays an important role in the regulation of mucus secretion in asthma patients [27]. In human airway epithelial cells, EGFR can be activated by oxidative stress. This in turn activates TNF-α–converting enzyme (TACE) which cleaves membrane-bound TGF-α to release the soluble cytokine, resulting in EGFR phosphorylation and expression of mucin genes such as MUC5AC and MUC5B [28]. Takeyama K *et al*. demonstrated that EGFR expression is increased in airway epithelial cells of asthma patients and that it is related to an increased expression of MUC5AC [29]. Sachdeva M *et al*. assumed that miR-145 was a specific cell type tumor suppressor which partially impacted metastasis and invasion by targeting mucin 1 [30]. TSLP is a cytokine that promotes CD4+ T cell homeostasis [31] and plays a critical role in asthma airway remodeling by inducing epithelium mesenchymal transformation [32]. In alleviated airway remodeling, TSLP is decreased. MMP-9 activation occurs in the inflamed airways [33], and Kin *et al*.'s study demonstrated that MMP-9 expression can be down-regulated by the EGFR inhibitor [34]. There is a known positive relationship between EGFR and MMP-9, therefore, decreased EGRF caused by miR-145 can lead to decreased MMP-9. TIMP-1 is a major endogenous inhibitor of MMP-9 [33]. It is reported that miR-145 can remarkably reduce MMP-9 and MMP-1 levels and slightly elevate TIMP-1 levels in J82 cells [35]. This is not in accordance with the results of the present study, therefore, future research is needed to confirm these results. There are existing studies that support the result that an elevation of IL-25 is caused by the transfection of miR-145 mimics and EGFR siRNA. However, this needs further exploration.

In our study, we found that mice in the asthma, asthma + miR-145 mimics NC and asthma + si-*EGFR* NC groups showed higher inflammatory cell infiltration, goblet cell hyperplasia and mucus obstruction. However, these conditions were remarkably alleviated in the asthma + miR-145 mimic and asthma + si-*EGFR* groups. This suggests that airway remodeling can be effectively treated by promoting miR-145 or silencing *EGFR*. Cytokines function is critical in chronic asthma inflammation as it recruits, activates and promotes the survival of multiple inflammatory cells of the respiratory tract [27]. Since asthma is characterized by chronic inflammation of the airways, miRNAs may play a role in its pathogenesis by modulating immune cells or responding to the regulation of structural cells such as epithelium or airway smooth muscle cells [36]. The asthma, asthma + miR-145 mimics NC and asthma + si-*EGFR* NC groups showed higher proportions of Th2 and Th17 cells in CD 4+ T cells of peripheral blood. There is increasing evidence which implicates the role of miRNAs in innate and acquired immune response by regulating the development, differentiation and function of immune cells (for example T-lymphocytes and B-lymphocytes) [37, 38]. Inflammatory response plays an important role in the progression and pathology of asthma as it involves the consistent recruitment of leukocytes (in particular eosinophils, Th2 and mast cells) [39, 40]. The EGFR pathway has been shown to have a critical role in airway dysfunction that is downstream of allergen induced inflammation and lung remodeling [14]. It either directly silences *EGFR* or leads to alleviated symptoms via miR-145.

In conclusion, miR-145 can decrease MUC5AC expression by inhibiting EGFR and alleviating airway remodeling. This indicates that miR-145 may be used as a molecular predictor for airway remodeling. However, we must also note that the collected samples size were limited. In future, a larger study is required to make the results of the present study more convincible. The study also showed that miR-145 causes a decreased level of TIMP-1. As this result cannot be supported by exiting studies, future studies should focus on exploring its specific mechanisms.

## MATERIALS AND METHODS

### Ethics statement

This study was approved by the Ethics Committee of the First Affiliated Hospital of Zhengzhou University and the methods used were carried out in accordance with the approved guidelines.

### Cell culture

Normal mouse alveolar epithelial cells (AECs) and asthmatic epithelial cells were purchased from the Chinese Academy of Sciences (Shanghai, China). Cells were inoculated in a medium (100 mm) (1×10^5^/mL). After adding Dulbecco's modified eagle's medium (DMEM, General Electric Company, Utah, USA) with 10% fetal bovine serum (FBS) (Gibco Company, Grand Island, NY, USA) the cells were cultured at 37°C with 5% CO_2_. Forty-eight hours later, the cells were treated with 0.25% trypsin (Biotime Biotechnology Co., Ltd. Shanghai, China) and re-cultured in a 75 mL flask. The culture medium was replaced every 3 days. Once 90% of the bottom of the flask was covered [41, 42], the cells were treated with 0.25% trypsin, centrifuged for 5 mins at 1000 rpm, the supernatant was removed, washed twice with DMEM and centrifuged again for 5 mins at 1000 rpm. The cells were suspended with serum-free DMEM and counted and diluted at 1×10^8^/mL.

### Dual luciferase reporter gene assay

DNA extraction was performed according to the operation instructions of the TIAN amp Genomic DNA Kit (TIANGEN Biotechnology Co. Ltd., Beijing, China). The vector psiCHECK-2-EGFR-3′UTR and a mutation vector psiCHECK-EGFR-Mut-3′UTR was constructed. AECs in the logarithmic growth phase were inoculated into a 6-well plate (4 × 10^3^/well) and cultured in an incubator at 37°C and with 5% CO_2_ for 24 hrs. The cells were transfected according to the Lipofectamine 2000 kit (Invitrogen Inc., Carlsbad, CA, USA) and divided into a WT + mimics (transfected with miR-145 mimics and EGFR-WT plasmids), MT + mimics (transfected with miR-145 mimics and EGFR-MT plasmids), WT + NC (transfected with mimic control and EGFR-WT plasmids) or a MT + NC group (transfected with mimic control and EGFR-MT plasmids). The transfection was performed four times in each group. The mimics and mimic control was purchased from Guangzhou RiboBio Co., Ltd. (Guangdong, China). Forty-eight hours after transfection a positive pyrolysis buffer was added to the cells of each group and mixed for 15 mins at room temperature. Subsequently, the supernatant was placed into a micro-well plate. Fluorescence values of each group were measured using the Thermo microplate reader (Thermo Fisher Scientific, California, USA). The value of substrate obtained after the reaction with firefly luciferase is represented by “F” while the measurement after the reaction with renilla luciferase is represented by “R”. Therefore, F/R represents relative luciferase activity.

### Cell grouping and transfection

Cells in the logarithmic growth phase were treated with 0.25% trypsin for 4 mins, centrifuged for 10 mins at 1000 × g and then suspended with DMEM. The cells were inoculated into a 12-well plate at 4 × 10^3^/well for 24 hrs. After the culture medium was removed, the cells were cultured in DMEM especially for experimental use for 24 hrs. Cells were then transfected according to the Lipofectamine 2000 (Invitrogen Inc., Carlsbad, CA, USA) instructions. The specific process was as follow: the miRNA and Lipofectamine 2000 reagent (100 μL) was independently diluted with serum-free DMEM and incubated for 5 mins at room temperature. The reagent was then quickly mixed to form a transfection complex (the total volume was 200 μL). Four hours after transfection, the primary culture medium was removed and the cells were cultured for 24 hrs in the transfection complex. The next day, the culture medium was replaced and the cells were re-cultured 48 hrs and small interference (siRNA) was used to interfere EGFR. The specific groupings were made before transfection: (1) control group; (2) blank group; (3) miR-145 mimics group; (4) mimic control group; (5) miR-145 inhibitors group; (6) inhibitor control group; (7) si-*EGFR* group and (8) the miR-145 inhibitor + si-*EGFR* group. Transfection was performed four times in each group. Normal alveolar epithelial cells (AEC) of mice in the control group received no treatment, while those in other groups were treated with the corresponding transfection. The miR-145 mimics, miR-145 inhibitors, corresponding mimic and inhibitor controls and si-*EGFR* were all purchased from Guangzhou RiboBio Co., Ltd. (Guangdong, China). After the culture medium replaced, cells were incubated for 48 hrs. Cells in logarithmic growth phase were selected for further experiments.

### Construction of lentivirus si-EGFR

Based on the known sequence design principles of GenBank *EGFR* (Gene number: NM_007312) and siRNA, we selected the primer sequences: siRNA, 5′-GCCTCCAGAGGATGTTCAA-3′ and negative 5′TAATCGTCGTAGACGGTTG-3′. The target fragment was inserted into the MluI and ClaI sites of the lentivirus plasmids vector pLVTHM. The lentivirus expression vectors LV-si-*EGFR* and siRNA NC were constructed with promoter H1 regulating siRNA expression and promoter EF1-α regulating green fluorescent protein (GFP).

### Establishment of mice model with chronic asthma

A total of 120 SPF-grade male BALB/c mice (6weeks old, weighing 20 ± 2 g) were purchased from the Shanghai SLAC Laboratory Animal Co., Ltd. (Shanghai, China). Mice were fed in a specific pathogen free (SPF)-grade environment at a temperature of 25°C and 70% humidity. Food and water was sterilized by ultraviolet light. Before the experiment, all mice were analyzed for normal lung functioning using the AniRes2005 mice lung function analysis system. All mice were confirmed to have normal lung function. After 2 weeks of adaptive feeding, the 120 mice were evenly divided into a normal, asthma, asthma + miR-145 mimics, asthma + miR-145 mimic NC, asthma + si-*EGFR* and asthma + si-*EGFR* NC group (Figure 6). In the asthma group, mice were intra-peritoneally injected with normal saline (0.2 mL) containing aluminum hydroxide gel (2 mg) (Aladdin, Shanghai, China) and ovalbumin (OVA) (50 μg) (Sigma-Aldrich Chemical Company, St Louis MO, USA) at 0 d, 7 d and 14 d [43]. At 21 d, 22 d and 23 d the mice were placed into an atomizer (KYWH1004, Foshan Turning Medical Technology Co., Ltd, Foshan, Guangdong, China) and those in the asthma, asthma + miR-145 mimics, asthma + miR-145 mimic NC, asthma + si-EGFR and asthma + si-EGFR NC groups were subjected to a phosphate buffered saline (PBS) solution with 1% OVA (30 min/time, 3 times/week× 5 weeks). The normal group inhaled a PBS solution rather than a OVA solution. Mice in the asthma group received no treatment. In the asthma + miR-145 mimics group, after inhaling an OVA solution and being anaesthetized the mice were given an intranasal instillation of lentivirusmiR-145 (5 × 107TU mL-1) (200 μL per mouse)(purchased from Guangzhou Ribobio Biotechnology Co., Ltd, Guangdong, China). Mice in the asthma + miR-145 mimic NC group inhaled an OVA solution and were given an intranasal instillation of equal-amount negative control lentivirus (the lentivirus vector LV included miR-145 and the negative control lentivirus vector with miR-145. The NC sequence was constructed with the help of Shanghai Genechem Co., Ltd., (Shanghai, China). The used lentiviral vector was LV-has plasmid). Intranasal instillation of lentivirus si-EGFR and the negative control lentivirus vector was independently given to the mice in the asthma + si-EGFR and asthma + si-EGFR NC groups after they inhaled the OVA solution. After these treatments all mice were sacrificed. The mice lung tissues were collected and independently fixed in a 10% formalin solution overnight. Part of the lung tissues was reserved in liquid nitrogen for further molecular biology experiments. All the above mentioned operations were conducted in accordance with the relevant provisions of the operation of experimental animals of the Institute of Clinical Medicine, from the First Affiliated Hospital of Zhengzhou University and approved by the Animal Ethics Association.

**Figure 6:** Procedure of mice model establishment and drug treatment. Note: miR-145, microRNA-145; NC, negative control; EGFR, epidermal growth factor receptor; PBS, phosphate buffer saline; OVA, ovalbumin.

### Hematoxylin and eosin (HE) and masson staining

The lung tissues were embedded overnight with paraffin and paraffin sections for HE and Masson staining. Following hematoxylin staining, tissues were washed with distilled water, washed with water in the wake of differentiation with hydrochloric acid, PBS anti-blue was applied and rewashed with water. The HE staining process was as follows: sections were stained with HE, treated with different levels of ethanol; treated with xylene three times and then mounted. The Masson staining process was as follows: stained with a ponceau-fuchsin solution, rinsed with glacial acetic acid and then immersed in phosphomolybdic acid. After the filter paper absorbed any excess liquid, the sections were stained with a aniline blue solution, immersed in glacial acetic acid, washing with water, air dried, treated with xylene three times and then mounted. Tissue morphology was observed under an electron microscope to determine whether the mice models with asthma were successively constructed and if there was any collagen deposition on related airway walls. With HE staining as a reference, the Image-Pro Plus 6.0 software was utilized to measure the perimeter of basement membrane (Pbm), total bronchial wall area (WAt), inner wall area (WAi), and smooth muscle wall area (WAm). These were all standardized using Pbm. The total Wat/Pbm, Wai/Pbm and WAm/Pbm were obtained to judge the degree of airway remodeling.

### Periodic acid-Schiff (PAS) staining

Lung tissues sections were de-waxed to water and first washed with 3% acetic acid for 2 mins and then a 1% Alcian blue-acetic acid solution was added and left for 10-20 mins. Subsequently, the sections were washed twice with distilled water for 5 mins each time. The tissues were immersed in a 0.5% periodic acid solution for 5 mins and then rewashed twice with distilled water (3 mins/time) and twice with 70% ethanol (3mins/time). Afterwards, the washed sections were immersed in Schiff solution for 15-30 mins and rewashed twice with flowing water (5 mins/time). Finally, sections were moderately stained with hematoxylin for 2-3 mins and any excess hematoxylin was rinsed off with flowing water. The section was then routinely de-waxed, covered with glass and sealed with neutral balsam. The lung histomorphology of each mice was observed under microscope (PAS staining kit was purchased from Sigma-Aldrich Chemical Company, St Louis MO, USA).

### Flow cytometry

The peripheral blood was obtained using eyeball extirpation. Following heparin treatment, the peripheral blood was mixed with monensin and then cultured in an incubator (50 mL/L CO_2_) at 37°C for 5 hrs. A total of 10 μL of anti-mouse mAb-anti-CD 4-FITC, anti-IL-4-PE, anti-IL-17-PE and isotype controls (Becton Dickinson Company, NJ, USA) was then added. The mixture was then incubated in the dark at room temperature for 30 mins, washed twice with PBS and suspended in 0.5 mL of PBS. Flow cytometer (purchased from Becton Dickinson Company, NJ, USA) was utilized for detection and Cell Quest software was used for data analysis.

### Enzyme-linked immune sorbent assay (ELISA)

Mice bronchial pulmonary alveolus was infused with bronchoalveolar lavage fluid (BALF), centrifuged at 1000 g for 5 mins and then the cell precipitation was re-suspended using 0.5 mL of PBS. Subsequently, 0.1 mL of the cells were placed on a blood-cell-counting plate to count the total number of cells. 0.2 mL of the cells were smeared and stained with Wright's. More than 200 cells were counted for classification. The supernatant was reserved for ELISA at -80°C. Tumor necrosis factor (TNF)-α, interleukin-4 (IL-4), IL-5, IL-13, IL-25, IL-33 and thymic stromal lymphopoietin (TSLP) in mice BALF was detected according to the ELISA kit (Shanghai Westang Biotechnology. Co., Ltd, Shanghai, China). Firstly, the kits were balanced for 20 mins at room temperature and a scrubbing solution was prepared. Ten standard wells were equipped on the ELISA plate (2 blank control groups were included with no sample or ELISA reagent). The standards received gradient dilution to make a standard curve. The samples to be tested were diluted and then placed into a well for microplate testing. After samples were gently mixed, the plate was sealed and cultured for 30 mins at 37°C. The liquid inside the well was removed, a scrubbing solution was added and then removed 30 secs later. This process was repeated 5 times followed by a spin dry. Afterwards, 50 μL of ELISA reagent was added to culture the samples for 30 mins at 37°C and then the liquid inside the well was removed. Subsequently, a scrubbing solution was added for 30mins and then removed. This process was repeated 5 times followed by a spin dry. In each well, 50 μL of development reagent A was first added and then 50 μL development reagent B was added. They were well mixed and cultured without light for 15 mins at 37°C. Finally, 50 μL of stop buffer was added. The blank control well was adjusted to be zero and the optical density (OD) value (450 nm) was measured within 15 mins using a microplate reader (Bio-Rad Laboratories, Inc., California, USA).

### Quantitative real-time polymerase chain reaction (qRT-PCR)

Total RNA of the cells and tissues were extracted using the TRIzol reagent. Reverse transcription of the extracted RNA was carried out using the TaqMan miRNA Reverse Transcription Kit (Applied Biosystems, Inc., CA, USA). The reaction conditions were 16°C for 30 mins, 42°C for 42 mins and 85°C for 5 mins. The TaqMan Universal PCR kit (Applied Biosystems, Inc., CA, USA) was utilized for qRT-PCR determination. The reaction volume was 20 μL; the reaction conditions were a warm start for 10 mins at 95°C, 15 secs at 95°C and 1 min at 60°C for a total of 40 cycles. ABI 7500 (Applied Biosystems, Inc., CA, USA) was applied for qRT-PCR. U6 was taken as a reference for miR-145 and glyceraldehyde-3-phosphate dehydrogenase (GAPDH) acted as a reference for EGFR, MUC5AC, TSLP, matrix metalloproteinase-9 (MMP-9) and tissue inhibitor of metalloproteinase-1 (TIMP-1). Related primer sequences are seen in Table 4. The data was analyzed using 2^−ΔΔCt^.

**Table 4:** Primer sequences for qRT-PCR

Primer	Sequence
miR-145	F: 5′-ATCGTCCAGTTTTCCCAGG-3′
	R: 5′-CGCCTCCACACACTCACC-3′
U6	F: 5′-ATTGGAACGATACAGAGAAGATT-3′
	R: 5′-GGAACGCTTCACGAATTTG-3′
EGFR	F: 5′-TCCCTCAGCCACCCATATGTAC-3′
	R: 5′-GTCTCGGGCCATTTTGGAGAATCC-3′
MUC5AC	F: 5′-GAGGGCAACAACGTCATCTCC-3′
	R: 5′-TCTTGGTCAGCCACCTTCACA-3′
TSLP	F: 5′-AAGTGCTACTAGTACGAGGTGG-3′
	R: 5′-CTTGGACTTGTGCCATTGAGCCT-3′
MMP-9	F: 5′-GGAGACCTGAGAACCAATCTC-3′
	R: 5′-TCCAATAGGTGATGTTGTCGT-3′
TIMP-1	F: 5′-CCTTCTGCAATTCCGACCTC-3′
	R: 5′-CGGGCAGGATTCAGGCTAT-3′
GAPDH	F: 5′-GCCGCATCTTCTTTTGCGTC-3′
	R: 5′-TACGACCAAATCCGTTGACTCC-3′

Note: miR-145, microRNA-145; qRT-PCR, quantitative real-time polymerase chain reaction; F, forward; R, reverse; EGFR, epidermal growth factor receptor; MUC5AC, mucin 5AC; TSLP, thymic stromal lymphopoietin; MMP-9, matrix metalloproteinase-9; TIMP-1, tissue inhibitor of metalloproteinase-1; GAPDH, glyceraldehyde-3-phosphate dehydrogenase.

### Western blotting

The miR-145-transfected cells and lung tissues in each group were washed with PBS and added to a cell lysis solution containing an appropriate amount of protease inhibitor. They were then shocked for 5 mins at 4°C, centrifugation (12000 ×g) for 10 mins at 4°C, the supernatant was collected, the Bradford method was used to measure the concentration of protein, 5 × loading buffer was added and then heated at 95°C for 10 mins. During the wet process, the upper sample (50 μg) was collected for sodium dodecyl sulfate polyacrylamide gel electrophoresis (SDS-PAGE) and then transferred to the cellulose nitrate membrane. After being sealed with milk, the sample was diluted with a Tween-20 (TBST) solution (1: 200) and incubated overnight with a *EGFR* monoclonal antibody (ab52894; 1: 1000; Abcam Inc., Cambridge, MA, USA), MU5AC (Rs-1022R; Shanghai Rui Qi Bio Technology Co., Ltd. Shanghai, China), TSLP (ab188766, 2.5 μg/mL, Abcam Inc., Cambridge, MA, USA), MMP-9 (ab38898; 1: 1000; Abcam Inc., Cambridge, MA, USA), TIMP-1 (ab1224; 1:500; Abcam Inc., Cambridge, MA, USA) and GAPDH (ab1224; 1: 500; Abcam Inc., Cambridge, MA, USA). The membrane was washed by TBST (4 × 10 min). After added with IRDyeTM 800DXlabelledIgG (diluted into 1: 10000), the protein sample was incubated for 1 h at room temperature. The membrane was washed with water four times and the substrate was added for developing. The protein bands were quantified using LabWorks Image Acquisition and Analysis Software (UVP, Inc., Upland, CA, USA).

### Statistical analysis

All data was analyzed using SPSS 19.0 statistic software (SPSS Inc., Chicago, IL, USA). Measurement data is expressed as $\bar{x}\pm s$. Before the analysis, the homogeneity of variance was analyzed and the normal distribution was tested. Comparison between the means of two samples with a normal distribution was verified using the *t* test. One-way analysis of variance (ANOVA) was used to validate comparison among groups. Comparison of the mean between groups was carried out using the LSD-*t* test. Bilateral *P* < 0.05 was considered to be statistically significant.

## References

[1] Akinbami LJ, Moorman JE, Bailey C, Zahran HS, King M, Johnson CA, Liu X (2012). Trends in asthma prevalence, health care use, and mortality in the United States, 2001-2010. NCHS Data Brief.

[2] Follenweider LM, Lambertino A (2013). Epidemiology of asthma in the United States. Nurs Clin North Am.

[3] Chen YH, Wu R, Geng B, Qi YF, Wang PP, Yao WZ, Tang CS (2009). Endogenous hydrogen sulfide reduces airway inflammation and remodeling in a rat model of asthma. Cytokine.

[4] Grainge CL, Lau LC, Ward JA, Dulay V, Lahiff G, Wilson S, Holgate S, Davies DE, Howarth PH (2011). Effect of bronchoconstriction on airway remodeling in asthma. N Engl J Med.

[5] Moffatt MF, Gut IG, Demenais F, Strachan DP, Bouzigon E, Heath S, von Mutius E, Farrall M, Lathrop M, Cookson WO, Consortium G (2010). A large-scale, consortium-based genomewide association study of asthma. N Engl J Med.

[6] Torgerson DG, Ampleford EJ, Chiu GY, Gauderman WJ, Gignoux CR, Graves PE, Himes BE, Levin AM, Mathias RA, Hancock DB, Baurley JW, Eng C, Stern DA (2011). Meta-analysis of genome-wide association studies of asthma in ethnically diverse North American populations. Nat Genet.

[7] Hassan T, McKiernan PJ, McElvaney NG, Cryan SA, Greene CM (2012). Therapeutic modulation of miRNA for the treatment of proinflammatory lung diseases. Expert Rev Anti Infect Ther.

[8] Liu Y, Sun X, Wu Y, Fang P, Shi H, Xu J, Li M (2015). Effects of miRNA-145 on airway smooth muscle cells function. Mol Cell Biochem.

[9] Perry MM, Adcock IM, Chung KF (2015). Role of microRNAs in allergic asthma: present and future. Curr Opin Allergy Clin Immunol.

[10] O'Leary L, Sevinc K, Papazoglou IM, Tildy B, Detillieux K, Halayko AJ, Chung KF, Perry MM (2016). Airway smooth muscle inflammation is regulated by microRNA-145 in COPD. FEBS Lett.

[11] Park SY, Roh SJ, Kim YN, Kim SZ, Park HS, Jang KY, Chung MJ, Kang MJ, Lee DG, Moon WS (2009). Expression of MUC1, MUC2, MUC5AC and MUC6 in cholangiocarcinoma: prognostic impact. Oncol Rep.

[12] Kanoh S, Tanabe T, Rubin BK (2011). IL-13-induced MUC5AC production and goblet cell differentiation is steroid resistant in human airway cells. Clin Exp Allergy.

[13] Ludovini V, Bellezza G, Pistola L, Bianconi F, Di Carlo L, Sidoni A, Semeraro A, Del Sordo R, Tofanetti FR, Mameli MG, Daddi G, Cavaliere A, Tonato M (2009). High coexpression of both insulin-like growth factor receptor-1 (IGFR-1) and epidermal growth factor receptor (EGFR) is associated with shorter disease-free survival in resected non-small-cell lung cancer patients. Ann Oncol.

[14] Hirota N, Risse PA, Novali M, McGovern T, Al-Alwan L, McCuaig S, Proud D, Hayden P, Hamid Q, Martin JG (2012). Histamine may induce airway remodeling through release of epidermal growth factor receptor ligands from bronchial epithelial cells. FASEB J.

[15] Guo YH, Gao FH, Shi J, Yuan HH, Jiang B (2013). [EGFR-ERK signaling pathway down-regulates miRNA-145 in lung cancer cells] [Article in Chinese]. Zhonghua Zhong Liu Za Zhi.

[16] Perrais M, Pigny P, Copin MC, Aubert JP, Van Seuningen I (2002). Induction of MUC2 and MUC5AC mucins by factors of the epidermal growth factor (EGF) family is mediated by EGF receptor/Ras/Raf/extracellular signal-regulated kinase cascade and Sp1. J Biol Chem.

[17] Bateman ED, Hurd SS, Barnes PJ, Bousquet J, Drazen JM, FitzGerald M, Gibson P, Ohta K, O'Byrne P, Pedersen SE, Pizzichini E, Sullivan SD, Wenzel SE (2008). Global strategy for asthma management and prevention: GINA executive summary. Eur Respir J.

[18] Cordes KR, Sheehy NT, White MP, Berry EC, Morton SU, Muth AN, Lee TH, Miano JM, Ivey KN, Srivastava D (2009). miR-145 and miR-143 regulate smooth muscle cell fate and plasticity. Nature.

[19] Uribe P, Gonzalez S (2011). Epidermal growth factor receptor (EGFR) and squamous cell carcinoma of the skin: molecular bases for EGFR-targeted therapy. Pathol Res Pract.

[20] Davies DE (2009). The role of the epithelium in airway remodeling in asthma. Proc Am Thorac Soc.

[21] Yoshikawa T, Kanazawa H, Tanaka J, Fujimoto S, Yamamoto T (2010). Gene polymorphism of epidermal growth factor receptor and airway hyperresponsiveness in young allergic subjects without respiratory symptoms. Med Sci Monit.

[22] Boxall C, Holgate ST, Davies DE (2006). The contribution of transforming growth factor-beta and epidermal growth factor signalling to airway remodelling in chronic asthma. Eur Respir J.

[23] Fedorov IA, Wilson SJ, Davies DE, Holgate ST (2005). Epithelial stress and structural remodelling in childhood asthma. Thorax.

[24] Polosa R, Puddicombe SM, Krishna MT, Tuck AB, Howarth PH, Holgate ST, Davies DE (2002). Expression of c-erbB receptors and ligands in the bronchial epithelium of asthmatic subjects. J Allergy Clin Immunol.

[25] Guo YH, Zhang C, Shi J, Xu MH, Liu F, Yuan HH, Wang JY, Jiang B, Gao FH (2014). Abnormal activation of the EGFR signaling pathway mediates the downregulation of miR145 through the ERK1/2 in non-small cell lung cancer. Oncol Rep.

[26] Cho WC, Chow AS, Au JS (2011). MiR-145 inhibits cell proliferation of human lung adenocarcinoma by targeting EGFR and NUDT1. RNA Biol.

[27] Barnes PJ (2008). The cytokine network in asthma and chronic obstructive pulmonary disease. J Clin Invest.

[28] Shao MX, Nadel JA (2005). Neutrophil elastase induces MUC5AC mucin production in human airway epithelial cells via a cascade involving protein kinase C, reactive oxygen species, and TNF-alpha-converting enzyme. J Immunol.

[29] Takeyama K, Fahy JV, Nadel JA (2001). Relationship of epidermal growth factor receptors to goblet cell production in human bronchi. Am J Respir Crit Care Med.

[30] Sachdeva M, Mo YY (2010). MicroRNA-145 suppresses cell invasion and metastasis by directly targeting mucin 1. Cancer Res.

[31] Al-Shami A, Spolski R, Kelly J, Keane-Myers A, Leonard WJ (2005). A role for TSLP in the development of inflammation in an asthma model. J Exp Med.

[32] Cho JY (2011). Recent advances in mechanisms and treatments of airway remodeling in asthma: a message from the bench side to the clinic. Korean J Intern Med.

[33] Ohbayashi H, Shimokata K (2005). Matrix metalloproteinase-9 and airway remodeling in asthma. Curr Drug Targets Inflamm Allergy.

[34] Kim S, Choi JH, Lim HI, Lee SK, Kim WW, Cho S, Kim JS, Kim JH, Choe JH, Nam SJ, Lee JE, Yang JH (2009). EGF-induced MMP-9 expression is mediated by the JAK3/ERK pathway, but not by the JAK3/STAT-3 pathway in a SKBR3 breast cancer cell line. Cell Signal.

[35] Kou B, Gao Y, Du C, Shi Q, Xu S, Wang CQ, Wang X, He D, Guo P (2014). miR-145 inhibits invasion of bladder cancer cells by targeting PAK1. Urol Oncol.

[36] Jiang X (2011). The emerging role of microRNAs in asthma. Mol Cell Biochem.

[37] Tsitsiou E, Lindsay MA (2009). microRNAs and the immune response. Curr Opin Pharmacol.

[38] Xiao C, Rajewsky K (2009). MicroRNA control in the immune system: basic principles. Cell.

[39] Sessa R, Hata A (2013). Role of microRNAs in lung development and pulmonary diseases. Pulm Circ.

[40] Frieri M (2007). Advances in the understanding of allergic asthma. Allergy Asthma Proc.

[41] Su F, Liu X, Liu G, Yu Y, Wang Y, Jin Y, Hu G, Hua S, Zhang Y (2013). Establishment and evaluation of a stable cattle type II alveolar epithelial cell line. PLoS One.

[42] Wang Y, Huang C, Reddy Chintagari N, Bhaskaran M, Weng T, Guo Y, Xiao X, Liu L (2013). miR-375 regulates rat alveolar epithelial cell trans-differentiation by inhibiting Wnt/beta-catenin pathway. Nucleic Acids Res.

[43] Fang C, Lu W, Li C, Peng X, Wang Y, Huang X, Yao Z, Cai N, Huang Y, Zhang X, Tan J (2016). MiR-3162-3p Is a Novel MicroRNA That Exacerbates Asthma by Regulating beta-Catenin. PLoS One.

